# Influence of *IGF2BP2, HMG20A*, and *HNF1B* genetic polymorphisms on the susceptibility to Type 2 diabetes mellitus in Chinese Han population

**DOI:** 10.1042/BSR20193955

**Published:** 2020-05-28

**Authors:** Ting Huang, Li Wang, Mei Bai, Jianwen Zheng, Dongya Yuan, Yongjun He, Yuhe Wang, Tianbo Jin, Wei Cui

**Affiliations:** 1 Nursing Department, The First Affiliated Hospital of Xi'an Jiaotong University. Xi’an 710061, China; 2 Key Laboratory of Molecular Mechanism and Intervention Research for Plateau Diseases of Tibet Autonomous Region, School of Medicine, Xizang Minzu University, Xianyang, Shaanxi 712082, China; 3 Department of Neurology, Affiliated hospital of Xizang Minzu University, Xianyang, Shaanxi 712082, China; 4 Department of Clinical Laboratory, Affiliated hospital of Xizang Minzu University, Xianyang, Shaanxi 712082, China; 5 Key Laboratory of Resource Biology and Biotechnology in Western China, Ministry of Education, School of Medicine, Northwest University, Xi’an 710069, Shaanxi, China; 6 Department of geriatric endocrinology, the First Affiliated Hospital of Xi'an Jiaotong University,Xi’an 710061,China

**Keywords:** Gene-behavioral habits, Polymorphism, Susceptibility, Type 2 diabetes mellitus

## Abstract

Background: The present study aimed to investigate the roles of insulin related gene *IGF2BP2, HMG20A*, and *HNF1B* variants in the susceptibility of Type 2 diabetes mellitus (T2DM), and to identify their association with age, gender, BMI, and smoking and alcohol drinking behavior among the Han Chinese population.

Methods: About 508 patients with T2DM and 503 healthy controls were enrolled. Rs11927381 and rs7640539 in *IGF2BP2*, rs7178572 in *HMG20A*, rs4430796, and rs11651052 in *HNF1B* were genotyped by using the Agena MassARRAY. Odds ratio (OR) and 95% confidence intervals (CI) were calculated by logistic regression.

Results: We found that *HMG20A* rs7178572 (OR = 1.25, *P* = 0.015) and *HNF1B* rs11651052 (OR = 1.26, *P* = 0.019) increased the risk of T2DM. Rs7178572, rs4430796, and rs11651052 might be related to the higher T2DM susceptibility not only by itself but also by interacting with age, gender smoking, and alcohol drinking. Rs11927381 also conferred the higher T2DM susceptibility at age ≤ 59 years. Besides, rs7178572-AA (*P* = 0.032) genotype and rs11651052 GG (*P* = 0.018) genotype were related to higher glycated hemoglobin and insulin level, respectively.

Conclusion: Specifically, we first found that rs11927381, rs7640539, and rs11651052 were associated with risk of T2DM among the Han Chinese population. We also provide evidence that age, gender, BMI, smoking, and drinking status have an interactive effect with these variants on T2DM susceptibility.

## Introduction

Type 2 diabetes mellitus (T2DM) is a complex, heterogeneous and chronic metabolic disorder, and is characterized by defects in insulin secretion and/or insulin action leading to hyperglycemia [1]. It is reported that about 1 in 11 adults have diabetes mellitus worldwide, 90% of whom have T2DM [2]. International Diabetes Federation Diabetes Atlas 2015 reported that China ranked first in the world for its population of diabetics. In China, the prevalence of T2DM was 9.6% in 2013, and was predicted to reach 13.0% in 2035 [3]. Numerous risk factors have been identified as potential contributors to T2DM susceptibility, such as physical activity, poor dietary condition, increasing obesity, aging, and genetic factors [4]. Recent studies suggested that genetic variants were considered to play a key role in the genesis of T2DM [5,6].

Insulin deficiency is the main characteristic of T2DM. Expression dysregulation of *IGF2BP2, HMG20A*, and *HNF1B* genes might affect the level of insulin and lead to the development of T2DM. *IGF2BP2* regulates insulin-like growth factor 2 (IGF2) translation that participates in the growth and insulin signaling pathways [7]. *HMG20A* is expressed in both human and mouse islets, and the levels of *HMG20A* are decreased in islets of T2DM donors compared with islets from non-diabetic donors [8]. *HNF1B* contributes to pancreatic cell formation and controls the specification, growth, and differentiation of the embryonic pancreas [9]. Although some studies have reported the relationship between *IGF2BP2, HMG20A*, and *HNF1B* polymorphisms and T2DM risk, the study on other polymorphisms in these genes is insufficient [10–12].

In the present study, we aimed to investigate the association of *IGF2BP2* rs11927381 and rs7640539, *HMG20A* rs7178572, *HNF1B* rs4430796, and rs11651052 variants with T2DM susceptibility among the Chinese Han population. Given that environment/lifestyle changes can modify the risk of T2DM [13], such as age, gender, body mass index (BMI), and smoking and alcohol drinking behavior, it is interesting to investigate whether these factors have an interactive effect with these variants on T2DM susceptibility.

## Subjects and methods

### Study participants

About 508 T2DM patients and 503 age- and gender-matched healthy controls were enrolled into the study from the First Affiliated Hospital of Xi’an Jiaotong University and Xizang Minzu University. All recruited subjects were genetically unrelated ethnic Han Chinese. T2DM cases were identified according to 2017 China Guideline for Type 2 Diabetes. T2DM patients were diagnosed as fasting plasma glucose ≥ 7.0 mmol/l and/or postprandial plasma glucose ≥11.1 mmol/l [14]. Patients who had Type 1 diabetes mellitus, gestational diabetes, acute or other chronic diseases, endocrine disorders, inflammatory diseases, or malignancy were excluded. The inclusion criteria for controls were with normal blood glucose levels and without family history of T2DM and no other chronic diseases. Demographic characteristics and clinical information were collected via standardized questionnaires and medical records. The data included age, sex, BMI, smoking, alcohol drinking, total cholesterol, high-density lipoprotein cholesterol (HDL-C), low-density lipoprotein cholesterol (LDL-C), serum uric acid, creatinine, glomerular filtration rate (GFR), fasting blood glucose, glycated hemoglobin, triglyceride, urea, creatinine, cystatin C, C-reactive protein, insulin, 25 hydroxy-vitamin D, ubiquitin cross-reactive protein (UCRP), and retinol-binding protein. The present study was approved by the ethics committee of Xizang Minzu University (201707) and was conducted in accordance with the declaration of Helsinki. All subjects signed an informed consent before enrolment in the study.

### Genotyping

Peripheral blood samples were obtained from each subject in vacutainers containing disodium-EDTA anticoagulant. Genomic DNA was isolated using the GoldMag DNA Purification Kit (GoldMag Co. Ltd, Xi′an, China) according to the manufacturer’s protocol, and was stored at −20°C until further analysis. Rs11927381 and rs7640539 in *IGF2BP2*, rs7178572 in *HMG20A*, rs4430796 and rs11651052 in *HNF1B* were selected according to the NCBI dbSNP database (http://www.ncbi.nlm.nih.gov/projects/SNP) and the 1000 Genomes Project data (http://www.internationalgenome.org/), with minor allele frequencies (MAFs) >5% and a pairwise tagging *r*^2^ of ≥0.8 in Chinese Han population. Genotyping was performed using Agena MassARRAY system (Agena, San Diego, CA, U.S.A.) [15,16], and conducted by two laboratory technicians in double-blind fashion. Primers for PCR amplification and single base extension were listed in Table 1. PCR products were sequenced with Agena MassARRAY Analyzer 4.0 software. Approximately 10% of samples were randomly selected to duplicate genotyping for quality control, and the concordance rates were 100%.

**Table 1:** Primers sequence of PCR and UEP used in the present study

Genes	SNPs	First primer (5′-3′)	Second primer (5′-3′)	UEP_DIR	UEP SEQ (5′-3′)
IGF2BP2	rs11927381	ACGTTGGATGAGTCTTATAGTAACTTGAG	ACGTTGGATGAGCCACAAGGAAACTTGATG	R	cCTTGAGATATTTTTGAAAGGTAAC
IGF2BP2	rs7640539	ACGTTGGATGCCAACCCAGATGATTTTGTC	ACGTTGGATGCACACCTGGCAGTGAAATTG	R	ggggAAATAGCACTGATACATTGTG
HMG20A	rs7178572	ACGTTGGATGCAACCTCATACCCAAAAATC	ACGTTGGATGGTATGGTTCAAGGTGAGTTG	R	ACCCAAAAATCTCTTACCA
HNF1B	rs4430796	ACGTTGGATGTGAATACAGAGAGGCAGCAC	ACGTTGGATGCAAAGACCCAACAACGCTTG	F	atGCAGCACAGACTGGA
HNF1B	rs11651052	ACGTTGGATGCCACCGTGTTCCCTTAAGAC	ACGTTGGATGTTCTCTTCCAGGAGGTTTAC	R	ccGTCGCGTTTTGGAGTTCC

Abbreviations: DIR, direction; SEQ, sequence; SNP, single-nucleotide polymorphism; UEP, unextended mini sequencing primer.

### Statistical analysis

Statistical analyses were carried out using SPSS version 17.0 (SPSS Inc., Chicago, IL, U.S.A.) and PLINK version 1.0.7. Demographic and clinical data between patients and controls were compared using chi-square test or independent sample *T* test, as appropriate. Continuous variables and categorical variables were presented as means ± standard deviation (SD) orabsolute number (percentage value), respectively. Hardy–Weinberg equilibrium (HWE) for each SNP in the control group was assessed using a goodness-of-fit χ^2^ test. The frequencies of genotype and allele between healthy controls and T2DM patients were compared with χ^2^ test. The correlation between selected SNPs and T2DM risk was estimated by odds ratios (OR) and 95% confidence intervals (CI) using logistic regression models, after adjusting for age and sex [17,18]. To explore the influence of gene–gene interactions on the risk of T2DM occurrence, multifactor dimensionality reduction (MDR) method was used [19]. Further, we stratified by gender, age, BMI, and behavioral factors (smoking and alcohol consumption) to adjust the possible cofounders. The associations of selected SNPs with the clinical parameters in T2DM patients were analyzed by one-way analysis of variance (ANOVA) test. A two-tailed *P* value < 0.05 was considered statistically significant.

## Results

About 508 patients with T2DM (59.21 ± 11.90 years, 277 males and 231 females) and 503 healthy controls (59.34 ± 7.62 years, 279 males and 224 females) were included. There was no significant differences in the distribution of age and gender between T2DM patients and the healthy controls (*P* = 0.841 and *P* = 0.712, respectively). Demographic and clinical characteristics of participants were listed in Table 2.

**Table 2:** Characteristics of patients with T2DM and controls

Variable	Cases (*n* = 508)	Controls (*n* = 503)	*P*
Age, year (mean ± SD)	59.21 ± 11.90	59.34 ± 7.62	0.841
>59	263 (51.8%)	265 (52.7%)	
≤59	245 (48.2%)	238 (47.3%)	
Gender			0.712
Male	277 (54.5%)	279 (55.5%)	
Female	231 (45.5%)	224 (44.5%)	
BMI (kg/m^2^)			
<24	130 (25.6%)	173 (34.4%)	
≥24	187 (36.8%)	185 (36.8%)	
Unavailable	191 (37.6%)	145 (28.8%)	
Smoking			
Yes	135 (26.6%)	115 (22.9%)	
No	230 (45.3%)	188 (37.4%)	
Unavailable	143 (28.1%)	200 (39.8%)	
Drinking			
Yes	68 (13.4%)	106 (21.1%)	
No	277 (54.5%)	182 (36.2%)	
Unavailable	163 (32.1%)	215 (42.7%)	
Total cholesterol (mmol/l)	4.61 ± 0.88	4.30 ± 1.63	**0.029**
HDL-C (mmol/l)	2.59 ± 0.75	2.49 ± 1.16	0.172
LDL-C (mmol/l)	1.12 ± 0.25	1.50 ± 7.45	0.378
Serum uric acid (μmol/l)	6.80 ± 19.8	5.96 ± 3.38	0.396
Creatinine (μmol/l)	67.85 ± 32.08	65.86 ± 32.18	0.390
GFR (ml/min)	95.95 ± 13.11	122.61 ± 35.88	**<0.001**
Fasting blood glucose	9.95 ± 4.70		
Glycated hemoglobin	9.30 ± 2.48		
Triglyceride	2.50 ± 2.26		
Urea	6.25 ± 3.19		
Creatinine	68.97 ± 29.49		
Cystatin C	0.97 ± 2.18		
Glomerular filtration rate	122.61 ± 35.88		
C-reactive protein	1.38 ± 1.57		
Insulin	18.80 ± 18.65		
25 hydroxy-vitamin D	24.69 ± 15.37		
UCRP	0.54 ± 1.28		
Retinol-binding protein	38.75 ± 11.14		

Abbreviations: BMI, body mass index; HDL-C, high-density lipoprotein cholesterol; LDL-C, low-density lipoprotein cholesterol; T2DM, Type 2 diabetes mellitus; UCRP, ubiquitin cross-reactive protein.

*P* values were calculated by χ^2^ test for continuous variables and Student’s *t* test for categorical variables.

Bold indicates that *P* < 0.05 means the data are statistically significant.

Five SNPs (rs11927381 and rs7640539 in *IGF2BP2*, rs7178572 in *HMG20A*, rs4430796, and rs11651052 in *HNF1B*) were successfully genotyped, and all SNPs were in accordance with HWE (*P* > 0.05, Table 3). The MAF of all SNPs was higher than 5% in T2DM patients and healthy controls. We also found the association of *HMG20A* rs7178572 and *HNF1B* rs11651052 with the increased T2DM susceptibility.

**Table 3:** The information about the candidate SNPs and associations with the risk of T2DM in allele model

Genes	SNPs ID	Chr: Position	Alleles	Frequency (MAF)		P^*^-value for HWE	OR (95%CI)	*P*^†^
			(Minor/Major)	Case	Control			
IGF2BP2	rs11927381	3:185790803	C/T	0.285	0.255	1.000	1.17 (0.96–1.42)	0.126
IGF2BP2	rs7640539	3:185795508	A/T	0.258	0.245	1.000	1.07 (0.88–1.31)	0.490
HMG20A	rs7178572	15:77454848	G/A	0.419	0.366	0.773	1.25 (1.04–1.49)	**0.015**
HNF1B	rs4430796	17:37738049	G/A	0.323	0.289	0.745	1.17 (0.97–1.42)	0.102
HNF1B	rs11651052	17:37742390	A/G	0.329	0.281	0.582	1.26 (1.04–1.52)	**0.019**

Abbreviations: HWE, Hardy–Weinberg equilibrium; MAF, minor allele frequency; SNP, single-nucleotide polymorphism; T2DM, Type 2 diabetes mellitus.

P^*^ for HWE values were calculated by χ^2^ test.

*P*^†^ values were calculated by logistic regression analysis with adjustments for age and gender.

Bold indicates that *P* < 0.05 means the data are statistically significant.

The genotype distribution for these SNPs and their relationship with T2DM susceptibility were shown in Table 4. For *HMG20A* rs7178572, the higher risk of T2DM occurrence was identified in genotype, dominant, and additive models. Besides, we found that *HNF1B* rs11651052 variant had an increased risk of T2DM in dominant and additive models.

**Table 4:** Relationships between *HMG20A* and *HNF1B* polymorphisms and T2DM risk

Genes	SNP ID	Model	Genotype	Case	Control	Adjusted by age and gender	
						OR (95%CI)	*p*
HMG20A	rs7178572	Genotype	AA	168	204	1	
			AG	257	230	1.36 (1.03–1.78)	**0.028**
			GG	85	69	1.50 (1.03–2.18)	**0.037**
		Dominant	AA	168	204	1	
			AG-GG	342	299	1.39 (1.07–1.79)	**0.012**
		Recessive	AA-AG	425	434	1	
			GG	85	69	1.26 (0.89–1.78)	0.192
		Log-additive	—			1.25 (1.05–1.50)	**0.015**
HNF1B	rs11651052	Genotype	GG	224	257	1	
			AG	236	209	1.30 (1.00–1.68)	0.050
			AA	50	37	1.55 (0.98–2.46)	0.062
		Dominant	GG	224	257	1	
			AA-AG	286	246	1.33 (1.04–1.71)	**0.023**
		Recessive	AG-GG	460	466	1	
			AA	50	37	1.37 (0.88–2.14)	0.165
		Log-additive	—			1.27 (1.04–1.54)	**0.017**

Abbreviations: 95%CI, 95% confidence interval; OR, odds ratio; SNP, single-nucleotide polymorphism; T2DM, Type 2 diabetes mellitus.

*P* values were calculated by logistic regression analysis with adjustments for age and gender.

Bold indicates that *P* < 0.05 means the data are statistically significant.

We further analyzed whether the genotypic effects on T2DM were dependent on gender and age (Table 5). We found that *HMG20A* rs7178572, *HNF1B* rs4430796, and rs11651052 were associated with the elevated T2DM susceptibility, especially in males. We found that individuals carrying rs7178572 G allele had an increased T2DM susceptibility under allele, homozygote, heterozygote, dominant, and additive models among males. Rs4430796 polymorphism contributed the risk of T2DM occurrence under allele, homozygote, recessive, and additive models among the male population. Rs11651052 variant was also a risk factor for T2DM among males under allele, homozygote, heterozygote, dominant, recessive, and additive models. Stratified by age, rs11927381, rs7178572, rs4430796, and rs11651052 were associated with the susceptibility to T2DM at age ≤59 years under multiple genetic models (Table 5). In the allele model, rs11927381, rs7178572, and rs11651052 were related to the elevated risk for T2DM. In the homozygote model, rs11927381, rs4430796, and rs11651052 conferred T2DM susceptibility. In the dominant model, rs11927381, rs7178572, and rs11651052 increased T2DM risk. In the recessive model, rs11927381 and rs11651052 had a higher susceptibility for T2DM. In the additive model, rs11927381, rs7178572, rs4430796, and rs11651052 contributed the developing of T2DM. However, there was a no significant relationship between these variants and T2DM among females or subjects with age >59 years.

**Table 5:** Relationships between *IGF2BP2, HMG20A*, and *HNF1B* polymorphisms and T2DM risk according to the stratification by gender and age

SNP ID	Model	Male		Female		>59 years		≤59 years	
		OR (95%CI)	*P*	OR (95%CI)	*P*	OR (95%CI)	*P*	OR (95%CI)	*P*
rs11927381	Allele	1.29 (0.99–1.68)	0.061	1.03 (0.77–1.39)	0.828	1.00 (0.76–1.30)	0.976	1.41 (1.06–1.89)	**0.020**
	Homozygote	1.66 (0.82–3.34)	0.159	1.30 (0.66–2.55)	0.445	0.96 (0.49–1.88)	0.910	2.65 (1.15–6.10)	**0.022**
	Heterozygote	1.32 (0.93–1.88)	0.114	0.89 (0.60–1.32)	0.559	1.10 (0.75–1.60)	0.633	1.36 (0.92–2.03)	0.127
	Dominant	1.36 (0.98–1.91)	0.069	0.96 (0.66–1.39)	0.824	1.07 (0.75–1.54)	0.704	1.50 (1.03–2.19)	**0.036**
	Recessive	1.46 (0.74–2.90)	0.277	1.36 (0.71–2.63)	0.357	0.92 (0.48–1.76)	0.810	2.35 (1.04–5.32)	**0.041**
	Additive	1.31 (0.99–1.72)	0.056	1.03 (0.78–1.37)	0.815	1.03 (0.78–1.36)	0.848	1.49 (1.09–2.03)	**0.012**
rs7178572	Allele	1.35 (1.06–1.72)	**0.015**	1.14 (0.88–1.49)	0.330	1.17 (0.91–1.49)	0.219	1.36 (1.05–1.76)	**0.021**
	Homozygote	1.74 (1.05–2.91)	**0.033**	1.26 (0.72–2.21)	0.424	1.40 (0.83–2.37)	0.205	1.66 (0.91–3.01)	0.098
	Heterozygote	1.46 (1.01–2.10)	**0.044**	1.25 (0.83–1.87)	0.284	1.22 (0.83–1.82)	0.314	1.50 (1.00–2.25)	0.050
	Dominant	1.52 (1.08–2.15)	**0.017**	1.25 (0.85–1.84)	0.255	1.27 (0.88–1.84)	0.208	1.53 (1.04–2.25)	**0.030**
	Recessive	1.42 (0.89–2.26)	0.147	1.11 (0.66–1.84)	0.701	1.25 (0.78–2.01)	0.355	1.32 (0.76–2.29)	0.324
	Additive	1.35 (1.06–1.72)	**0.016**	1.15 (0.88–1.50)	0.318	1.19 (0.92–1.54)	0.176	1.34 (1.01–1.77)	**0.040**
rs4430796	Allele	1.33 (1.03–1.72)	**0.027**	0.99 (0.74–1.32)	0.943	1.07 (0.82–1.40)	0.600	1.28 (0.97–1.68)	0.079
	Homozygote	2.09 (1.12–3.92)	**0.021**	0.94 (0.49–1.80)	0.848	1.37 (0.72–2.58)	0.336	2.10 (1.06–4.17)	**0.034**
	Heterozygote	1.23 (0.86–1.74)	0.252	1.02 (0.69–1.51)	0.914	1.09 (0.75–1.59)	0.655	1.22 (0.83–1.81)	0.313
	Dominant	1.34 (0.96–1.87)	0.087	1.01 (0.70–1.45)	0.977	1.14 (0.80–1.62)	0.484	1.34 (0.92–1.95)	0.124
	Recessive	1.89 (1.04–3.46)	**0.038**	0.93 (0.50–1.74)	0.819	1.31 (0.71–2.42)	0.382	1.90 (0.98–3.67)	0.056
	Additive	1.35 (1.04–1.75)	**0.024**	0.99 (0.75–1.31)	0.936	1.14 (0.87–1.49)	0.355	1.35 (1.01–1.81)	**0.041**
rs11651052	Allele	1.47 (1.14–1.89)	**0.003**	1.03 (0.78–1.37)	0.840	1.16 (0.89–1.51)	0.274	1.35 (1.03–1.78)	**0.029**
	Homozygote	2.47 (1.29–4.73)	**0.007**	0.93 (0.47–1.82)	0.823	1.29 (0.67–2.49)	0.452	2.32 (1.15–4.70)	**0.019**
	Heterozygote	1.43 (1.01–2.02)	**0.047**	1.14 (0.77–1.67)	0.522	1.25 (0.86–1.81)	0.244	1.38 (0.93–2.05)	0.106
	Dominant	1.55 (1.11–2.17)	**0.010**	1.10 (0.76–1.58)	0.627	1.26 (0.88–1.79)	0.211	1.50 (1.03–2.18)	**0.035**
	Recessive	2.07 (1.11–3.88)	**0.023**	0.87 (0.46–1.67)	0.684	1.17 (0.62–2.20)	0.639	1.97 (1.02–3.87)	**0.049**
	Additive	1.50 (1.15–1.96)	**0.003**	1.03 (0.77–1.37)	0.844	1.18 (0.9–1.56)	0.239	1.46 (1.09–1.97)	**0.012**

Abbreviations: 95%CI, 95% confidence interval; OR, odds ratio; SNP, single-nucleotide polymorphism; T2DM, Type 2 diabetes mellitus.

*P* values were calculated by logistic regression analysis with adjustments for age and gender.

Bold indicates that *P* < 0.05 means the data are statistically significant.

Stratified analyses were also carried out to estimate the effect of these polymorphisms with BMI and behavioral factors (smoking and alcohol consumption) on T2DM risk, as shown in Table 6. For rs7178572 variant, the G allele carriers had an increased risk of T2DM occurrence among subjects with BMI > 24 kg/m^2^ (allele, homozygote, and recessive), smokers (allele, homozygote, and recessive), or alcohol drinkers (homozygote and recessive). For rs4430796 polymorphism, GG genotype was predominantly related to a higher risk of T2DM among subjects with BMI ≤ 24 kg/m^2^ or drinkers. Besides, rs4430796 also showed a risk-increasing effect among non-drinkers. For rs11651052 variant, BMI, smoking, and alcohol drinking status had interactive effect with selected SNPs on T2DM risk. An association of rs11651052 and T2DM risk was observed in both subjects with BMI > 24 kg/m^2^ (allele, dominant, and additive) and subjects BMI ≤ 24 kg/m^2^ (homozygote and additive). In non-smokers, a trend of higher risk of developing T2DM was also found for subjects with A allele, and AA, AA-AG genotypes, and in additive model. Similarly, rs11651052-A allele had a higher the incidence of T2DM in smokers. In drinkers, individuals with rs11651052 AA genotype had 7.65- and 7.49-fold increased risk of developing T2DM than drinkers who carried GG genotype and combined AG-GG, respectively. In non-drinkers, rs11651052 was also associated with T2DM occurrence (allele, dominant, and additive).

**Table 6:** Relationships between *IGF2BP2, HMG20A*, and *HNF1B* polymorphisms and T2DM risk according to the stratification by BMI, smoking, and drinking

SNP ID	Model	BMI > 24 kg/m^2^		BMI ≤ 24 kg/m^2^		Smoking		Non-smoking		Alcohol drinking		Not alcohol drinking	
		OR (95%CI)	*P*	OR (95%CI)	*P*	OR (95%CI)	*P*	OR (95%CI)	*P*	OR (95%CI)	*P*	OR (95%CI)	*P*
rs7178572	Allele	1.54 (1.15–2.07)	**0.004**	0.99 (0.71–1.38)	0.966	1.55 (1.08–2.22)	**0.017**	1.04 (0.78–1.37)	0.795	1.40 (0.90–2.18)	0.134	1.13 (0.86–1.48)	0.369
	Homozygote	2.71 (1.12–6.54)	**0.027**	0.92 (0.40–2.10)	0.839	3.32 (1.10–10.01)	**0.034**	1.12 (0.57–2.19)	0.746	3.37 (1.05–10.76)	**0.041**	1.09 (0.57–2.09)	0.801
	Heterozygote	1.00 (0.58–1.73)	0.999	1.41 (0.81–2.45)	0.227	1.07 (0.50–2.28)	0.869	1.22 (0.77–1.91)	0.396	0.71 (0.31–1.60)	0.406	1.30 (0.83–2.03)	0.247
	Dominant	1.20 (0.71–2.04)	0.499	1.29 (0.76–2.19)	0.348	1.38 (0.67–2.84)	0.387	1.20 (0.78–1.84)	0.418	1.03 (0.48–2.19)	0.948	1.25 (0.82–1.92)	0.297
	Recessive	2.71 (1.20–6.09)	**0.016**	0.76 (0.35–1.63)	0.473	3.19 (1.17–8.70)	**0.024**	1.00 (0.54–1.86)	1.000	4.12 (1.42–11.95)	**0.009**	0.93 (0.51–1.69)	0.808
	Additive	1.42 (0.97–2.09)	0.072	1.07 (0.73–1.56)	0.747	1.62 (0.97–2.70)	0.063	1.10 (0.80–1.51)	0.557	1.51 (0.88–2.58)	0.137	1.11 (0.81–1.51)	0.528
rs4430796	Allele	1.34 (0.98–1.83)	0.067	1.27 (0.89–1.80)	0.188	1.41 (0.96–2.07)	0.082	1.33 (0.99–1.79)	0.062	1.45 (0.91–2.30)	0.117	1.35 (1.01–1.81)	**0.044**
	Homozygote	1.76 (0.71–4.32)	0.221	4.23 (1.12–16.02)	**0.034**	4.46 (0.86–23.24)	0.076	2.05 (0.89–4.74)	0.093	7.96 (1.31–48.51)	**0.025**	1.75 (0.78–3.91)	0.174
	Heterozygote	1.34 (0.79–2.26)	0.274	1.19 (0.70–2.02)	0.518	0.88 (0.44–1.77)	0.720	1.35 (0.87–2.10)	0.179	0.70 (0.32–1.52)	0.368	1.39 (0.91–2.13)	0.127
	Dominant	1.41 (0.86–2.31)	0.178	1.35 (0.81–2.26)	0.249	1.07 (0.55–2.09)	0.842	1.44 (0.94–2.20)	0.090	0.97 (0.47–2.01)	0.940	1.44 (0.96–2.17)	0.079
	Recessive	1.53 (0.64–3.66)	0.335	3.88 (1.05–14.32)	**0.042**	4.73 (0.94–23.85)	0.060	1.78 (0.79–4.00)	0.165	9.39 (1.60–55.05)	**0.013**	1.50 (0.68–3.27)	0.313
	Additive	1.33 (0.91–1.95)	0.144	1.49 (0.97–2.29)	0.072	1.32 (0.77–2.27)	0.316	1.39 (1.00–1.95)	0.053	1.41 (0.78–2.52)	0.253	1.36 (0.98–1.88)	0.070
rs11651052	Allele	1.51 (1.11–2.07)	**0.010**	1.27 (0.90–1.80)	0.174	1.51 (1.02–2.23)	**0.039**	1.40 (1.04–1.89)	**0.026**	1.56 (0.98–2.46)	0.058	1.43 (1.07–1.92)	**0.015**
	Homozygote	2.44 (0.97–6.13)	0.058	3.41 (1.00–11.59)	**0.049**	5.01 (0.96–26.05)	0.056	2.35 (1.02–5.40)	**0.044**	7.65 (1.40–41.85)	**0.019**	1.98 (0.89–4.41)	0.093
	Heterozygote	1.54 (0.91–2.61)	0.109	1.44 (0.84–2.45)	0.183	1.14 (0.57–2.28)	0.711	1.48 (0.95–2.30)	0.084	1.04 (0.48–2.26)	0.924	1.49 (0.97–2.28)	0.069
	Dominant	1.68 (1.02–2.77)	**0.043**	1.57 (0.94–2.65)	0.087	1.35 (0.69–2.64)	0.376	1.59 (1.04–2.44)	**0.032**	1.35 (0.64–2.84)	0.426	1.56 (1.03–2.34)	**0.034**
	Recessive	1.99 (0.82–4.84)	0.128	2.83 (0.86–9.30)	0.087	4.7 (0.94–23.57)	0.060	1.95 (0.87–4.35)	0.104	7.49 (1.44–39.00)	**0.017**	1.65 (0.76–3.57)	0.208
	Additive	1.55 (1.05–2.29)	**0.026**	1.60 (1.03–2.48)	**0.035**	1.54 (0.89–2.67)	0.122	1.51 (1.08–2.12)	**0.017**	1.72 (0.95–3.13)	0.075	1.44 (1.04–2.00)	**0.028**

Abbreviations: 95%CI, 95% confidence interval; BMI, body mass index; OR, odds ratio; SNP, single nucleotide polymorphism; T2DM, Type 2 diabetes mellitus.

*P* values were calculated by logistic regression analysis with adjustments for age and gender.

Bold indicates that *P* < 0.05 means the data are statistically significant.

The association between higher order interactions of SNP–SNP and T2DM risk was analyzed by MDR as summarized in Figure 1. The interaction analysis revealed moderate effect between the markers *HMG20A* rs7178572, *HNF1B* rs11651052, and *IGF2BP2* rs7640539, which were conferring risk toward T2DM progression. The accumulated effect of rs7178572-GG, rs11651052-AA, and rs7640539-TA conferred a higher risk for T2DM, as shown in Table 7.

**Figure 1:** Summary of MDR SNP–SNP interaction among *IGF2BP2, HMG20A*, and *HNF1B* gene Dark-shaded cells represent higher risk combinations compared with light-shaded cells. Each cell shows counts of “case” on left and “control” on right.

**Table 7:** SNP–SNP interaction models of the *IGF2BP2, HMG20A*, and *HNF1B* genes analyzed by the MDR method

Model	Training Bal. Acc.	Testing Bal. Acc.	CVC	OR (95%CI)	*P*
*HMG20A* rs7178572	0.539	0.531	9/10	1.46 (1.12–1.91)	**0.0058**
*HMG20A* rs7178572, *HNF1B* rs11651052	0.550	0.510	7/10	1.63 (1.25–2.15)	**0.0004**
*HMG20A* rs7178572, *HNF1B* rs11651052 and *IGF2BP2* rs7640539	0.574	0.524	6/10	1.89 (1.45–2.48)	**<0.0001**

Bal. Acc., balanced accuracy; CI, confidence interval; CVC, cross–validation consistency; MDR, multifactor dimensionality reduction; OR, odds ratio.

*P* values were calculated using χ^2^ tests.

Bold indicates that *P* < 0.05 means the data are statistically significant.

The relation between selected SNPs and different clinical parameters of T2DM patients was investigated, as illustrated in Table 8. We found the significant relationship of *IGF2BP2* rs11927381 and rs7640539 with the levels of retinol-binding protein (*P* = 0.010 and *P* = 0.028, respectively). The association of *HMG20A* rs7178572 with glycated hemoglobin was identified (*P* = 0.032). Besides, carriers of *HNF1B* rs11651052 GG genotype had significantly higher insulin level than AA and AG genotypes (*P* = 0.018). However, there was no relation of different genotypes with the remaining clinical parameters (*P* > 0.05).

**Table 8:** Comparisons of clinical characteristics among T2DM patients with different genotypes of SNPs in *IGF2BP2, HMG20A*, and *HNF1B*

Characteristics	rs11927381				rs7640539			
	TT	CT	CC	*P*	AA	AT	TT	*P*
Total cholesterol	4.53 ± 1.36	4.49 ± 1.31	4.72 ± 1.05	0.650	4.65 ± 1.10	4.51 ± 1.29	4.52 ± 1.36	0.876
HDL-C	1.19 ± 0.58	1.18 ± 0.50	1.34 ± 0.87	0.314	1.37 ± 0.95	1.18 ± 0.50	1.19 ± 0.56	0.258
LDL-C	2.70 ± 1.14	2.55 ± 0.96	2.50 ± 0.79	0.306	2.44 ± 0.83	2.56 ± 0.95	2.67 ± 1.11	0.376
Urea	6.35 ± 2.95	5.98 ± 1.91	6.77 ± 6.93	0.317	7.22 ± 7.61	6.00 ± 1.94	6.29 ± 2.87	0.155
Creatinine	70.67 ± 35.71	68.25 ± 22.19	63.15 ± 18.29	0.336	63.49 ± 19.43	68.03 ± 22.68	70.41 ± 34.39	0.425
Glomerular filtration rate	124.44 ± 36.99	121.03 ± 32.41	123.58 ± 37.93	0.737	123.59 ± 39.83	121.48 ± 33.00	124.03 ± 36.32	0.845
Fasting blood glucose	9.51 ± 3.59	10.51 ± 5.92	9.80 ± 4.06	0.196	9.69 ± 4.18	10.65 ± 6.06	9.53 ± 3.55	0.135
Glycated hemoglobin	9.16 ± 2.08	9.39 ± 2.90	9.49 ± 2.45	0.672	9.63 ± 2.40	9.41 ± 2.98	9.18 ± 2.10	0.604
Triglyceride	2.60 ± 2.47	2.35 ± 1.86	2.61 ± 2.79	0.646	2.75 ± 2.88	2.29 ± 1.72	2.60 ± 2.50	0.456
Cystatin C	0.88 ± 0.54	0.81 ± 0.19	0.80 ± 0.33	0.340	0.79 ± 0.35	0.80 ± 0.19	0.88 ± 0.52	0.289
C-reactive protein	1.40 ± 0.97	1.38 ± 2.19	1.11 ± 0.85	0.708	1.11 ± 0.87	1.39 ± 2.27	1.40 ± 0.96	0.721
Insulin	19.83 ± 21.28	17.30 ± 16.05	18.21 ± 10.35	0.553	18.54 ± 10.49	17.49 ± 16.52	19.76 ± 20.74	0.631
25-Hydroxy-vitamin D	25.77 ± 16.79	23.25 ± 14.28	24.74 ± 9.11	0.521	24.95 ± 9.37	23.02 ± 14.77	25.68 ± 16.36	0.494
UCRP	0.46 ± 1.17	0.67 ± 1.49	0.43 ± 0.56	0.353	0.46 ± 0.57	0.67 ± 1.49	0.47 ± 1.18	0.414
Retinol-binding protein	40.65 ± 11.13	36.01 ± 10.60	38.12 ± 9.47	**0.010**	37.54 ± 9.42	36.26 ± 10.69	40.44 ± 11.42	**0.028**

Characteristics	rs7178572				rs11651052			
	AA	GA	GG	*P*	AA	AG	GG	*P*
Total cholesterol	4.48 ± 1.18	4.59 ± 1.46	4.46 ± 1.10	0.660	4.67 ± 1.11	4.46 ± 1.33	4.59 ± 1.35	0.527
HDL-C	1.16 ± 0.51	1.21 ± 0.60	1.26 ± 0.63	0.501	1.15 ± 0.35	1.23 ± 0.66	1.18 ± 0.51	0.628
LDL-C	2.54 ± 0.88	2.66 ± 1.07	2.65 ± 1.24	0.611	2.85 ± 1.18	2.61 ± 1.11	2.57 ± 0.92	0.308
Urea	6.48 ± 4.15	6.28 ± 2.84	5.66 ± 1.63	0.237	6.07 ± 1.92	6.01 ± 2.90	6.55 ± 3.69	0.260
Creatinine	67.87 ± 35.06	69.64 ± 27.23	69.15 ± 23.39	0.864	67.53 ± 25.05	69.59 ± 36.58	68.61 ± 20.27	0.902
Glomerular filtration rate	124.6 ± 41.72	123.06 ± 31.73	119.77 ± 32.46	0.754	123.84 ± 36.27	126.7 ± 36.07	118.56 ± 33.64	0.182
Fasting blood glucose	10.89 ± 5.79	9.52 ± 4.29	9.45 ± 3.07	0.051	9.54 ± 4.29	9.77 ± 4.14	10.27 ± 5.37	0.578
Glycated hemoglobin	9.84 ± 3.26	9.05 ± 2.01	9.01 ± 1.82	**0.032**	8.77 ± 2.31	9.18 ± 2.65	9.56 ± 2.30	0.206
Triglyceride	2.30 ± 1.70	2.64 ± 2.51	2.40 ± 2.37	0.470	2.52 ± 2.04	2.44 ± 2.23	2.56 ± 2.37	0.911
Cystatin C	0.81 ± 0.23	0.88 ± 0.55	0.83 ± 0.17	0.427	0.98 ± 1.10	0.82 ± 0.24	0.84 ± 0.22	0.164
C-reactive protein	1.17 ± 0.70	1.50 ± 2.03	1.41 ± 1.09	0.291	1.27 ± 0.83	1.24 ± 0.78	1.56 ± 2.25	0.257
Insulin	20.09 ± 23.45	17.80 ± 16.19	19.30 ± 14.80	0.643	15.26 ± 9.78	16.44 ± 15.14	22.55 ± 23.15	**0.018**
25-Hydroxy-vitamin D	25.17 ± 20.70	24.61 ± 12.56	23.87 ± 8.19	0.915	27.57 ± 21.20	25.43 ± 18.05	22.9 ± 7.85	0.319
UCRP	0.74 ± 1.73	0.42 ± 0.95	0.55 ± 1.15	0.162	0.32 ± 0.62	0.52 ± 1.34	0.63 ± 1.33	0.446
Retinol-binding protein	38.49 ± 10.21	38.99 ± 11.60	38.54 ± 11.77	0.948	37.70 ± 8.33	38.31 ± 11.11	39.55 ± 11.79	0.659

Abbreviations: HDL-C, high-density lipoprotein cholesterol; LDL-C, low-density lipoprotein cholesterol; SNP, single-nucleotide polymorphism; T2DM, Type 2 diabetes mellitus; UCRP, ubiquitin cross-reactive protein.

*P* values were calculated by using one-way analysis of variance (ANOVA) test.

Bold indicates that *P* < 0.05 means the data are statistically significant.

## Discussion

We performed a case–control study to investigate the association of *IGF2BP2* rs11927381 and rs7640539, *HMG20A* rs7178572, *HNF1B* rs4430796, and rs11651052 with T2DM susceptibility. We found that *HMG20A* rs7178572 and *HNF1B* rs11651052 were related to an increased T2DM risk in the overall. Given that T2DM represents a complex disorder influenced by the interplay between genetic and behavioral factors, we analyzed the effect of age, gender, BMI, smoking, and alcohol drinking on the relationship of these variants with T2DM susceptibility. Our stratified analysis showed that rs7178572, rs4430796, and rs11651052 had higher risk of T2DM occurrence in males and subjects with age ≤ 59 years. In addition, rs11927381 also contributed T2DM susceptibility at age ≤ 59 years. We also found that these genetic variants might increase the risk of T2DM occurrence not only by itself but also by interacting with smoking and alcohol drinking. Besides, rs7178572-AA (*P* = 0.032) genotype and rs11651052 GG (P = 0.018) genotype might have higher glycated hemoglobin and insulin levels, respectively. To the best of our knowledge, this was the first to explore the effects of the relationships between *IGF2BP2* rs11927381, rs7640539 and *HNF1B* rs11651052 and T2DM susceptibility in the Chinese Han population.

Insulin-like growth factor 2 binding protein 2 (*IGF2BP2*), located on chromosome 3q27, encodes an mRNA-binding protein associated with RNA location, stability, and translation. *IGF2BP2*, highly expressed in pancreatic islets, is involved in β-cell function by regulating IGF2 post-translational modification [20]. IGF2 is a member of the insulin family of polypeptide growth factors, which play an important role in the development, growth, and stimulation of insulin action [21]. *IGF2BP2* variations were also associated with decreased insulin secretion and hyperglycemia [22]. Several variants in *IGF2BP2* were investigated for the relationship with T2DM; however, there were very few studies on rs11927381 and rs7640539. Only one study reported the association between *IGF2BP2* rs11927381 and the increased T2DM risk among Slavonic population [23]. There was no report on rs7640539 polymorphism. Our results displayed rs11927381 variant had a higher risk of developing T2DM in subjects with age ≤ 59 years, suggesting the association appear to be age dependent. However, the current study did not find a significant relationship between rs7640539 and T2DM susceptibility. Further studies are required to elucidate the association.

High mobility group 20 A (*HMG20A*) gene, located in 15q24.3, is a member of high mobility group (HMG) box-containing genes. *HMG20A* encodes a widely expressed non-histone chromosomal protein controlling gene expression by histone modification [24].

*HMG20A* expression in islet is essential for metabolism-insulin secretion coupling via the coordinated regulation of key islet-enriched genes, and the depletion HMG20A protein induces expression of genes implicated in β cell de-differentiation [8]. Previously, *HMG20A* (rs7178572) showed an association with T2DM in European obese subjects [25]. Our results found that G allele of rs7178572, intronic SNPs within the *HMG20A*, which was related to an increased T2DM susceptibility. However, a previous study showed there was no significant relationship between rs7178572 and the risk of T2DM among Han population in southern China [26], such inconsistencies in these reports might result from a different behavioral habit or sample size. As we known, genetic, environmental, behavioral, and metabolic risk factors are contributed to the development of T2DM [27]. Obesity (defined by BMI), smoking, and alcohol drinking (especially heavy alcohol consumption) are known risk factors for T2DM [28–30]. Smoking increased 1.35-fold the risk of T2DM compared with non-smokers [29]. Alcohol consumption is related to glycemic control and insulin resistance [30]. Therefore, we evaluated the effects of age, gender, BMI, smoking, and alcohol consumption on the association of rs7178572 with T2DM risk. Interestingly, rs7178572 variant had a higher susceptibility to T2DM in males, smokers, drinkers, and the subjects with BMI > 24 kg/m^2^. These results are required to validate in larger populations.

Hepatocyte nuclear factor-1β (*HNF1B*), located on chromosome 17q21.3, encodes a transcription factor that involved in tissue-specific regulation of gene expression and embryonic development of numerous organs [31]. *HNF1B* gene played the important role in the primary pathophysiology of diabetes. It was involved in the loss of neurogenin-3 (Ngn3)-positive endocrine progenitor cells, pancreatic atrophy, and a reduced insulin sensitivity to endogenous glucose production leading to the reduction of insulin secretion [32]. Previous studies have reported that genetic variations in *HNF1B* were associated with the susceptibility of T2DM. Rs4430796 (A>G) in intron 2 of *HNF1B* is the most frequent SNP in Chinese population. Notably, the mutant allele frequency for rs4430796 is quite different between different ethnic groups. The mutant allele G frequency in the study was 0.289, similar to the healthy Han Chinese and Asian, but significantly different from Caucasian (0.47) and African (0.67) [33]. Previous studies revealed the risk G allele of rs4430796 was significantly related to T2DM in a southern Chinese Han population [34], which was consistent with our results. Here, we found that rs4430796 increased the risk of T2DM occurrence, especially in males and subgroup with age ≤ 59 years. Besides, the association also was observed in the subgroup with BMI ≤ 24 kg/m^2^ and drinkers. These results indicated that gene-behavioral habit interactions might operate in the pathogenesis of T2DM. Rs11651052 (G > A) is another SNP in *HNF1B*, and no study has analyzed the SNP now. In our study, we first reported that rs11651052-A allele increased 1.26-fold risk of T2DM compared with G allele. Our stratified analysis showed that rs11651052 had a higher T2DM susceptibility in males and subjects with age ≤ 59 years, suggesting the risk association of this polymorphism might be age dependent.

Inevitably, several intrinsic limitations should be considered. First, the subjects were enrolled from the identical hospitals; therefore, the selection bias could not be completely excluded. Second, some clinical characteristics were not analyzed because of missing or uncollected data in controls. Third, explicit mechanisms of these polymorphisms on the development of T2DM are still bewildered and further research is required. Therefore, further well-designed large and prospective studies and functional experiments should be conducted to verify our finding.

## Conclusion

To sum up, our study revealed that variants in *IGF2BP2, HMG20A*, and *HNF1B* had the risk effect on T2DM occurrence among the Chinese Han population. Specifically, we first found that rs11927381, rs7640539, and rs11651052 were associated with the increased risk of T2DM occurrence. We also provided evidence that age gender, BMI, smoking, and alcohol drinking status had interactive effect with these variants on T2DM susceptibility, suggesting that gene-behavioral habit interactions might play critical roles in the risk of developing T2DM. Our study may increase the understanding of *IGF2BP2, HMG20A*, and *HNF1B* variants on the pathogenesis of T2DM.

## Abbreviations

CI: confidence interval
CVC: cross–validation consistency
HDL-C: high-density lipoprotein cholesterol
HWE: Hardy–Weinberg equilibrium
IGF2: insulin-like growth factor 2
LDL-C: low-density lipoprotein cholesterol
MDR: multifactor dimensionality reduction
OR: odds ratio
SNP: single-nucleotide polymorphism
T2DM: Type 2 diabetes mellitus
